# Comparison of the Effectiveness of Water-Based Extraction of Substances from Dry Tea Leaves with the Use of Magnetic Field Assisted Extraction Techniques

**DOI:** 10.3390/molecules22101656

**Published:** 2017-10-03

**Authors:** Grzegorz Zaguła, Marcin Bajcar, Bogdan Saletnik, Maria Czernicka, Czesław Puchalski, Ireneusz Kapusta, Jan Oszmiański

**Affiliations:** 1 Department of Bioenergetics and Food Analysis, Faculty of Biology and Agriculture, University of Rzeszów, 35-601 Rzeszów, Poland; mbajcar@ur.edu.pl (M.B.); bogdan.saletnik@urz.pl (B.S.); mczernicka@ur.edu.pl (M.C.); cpuchal@ur.edu.pl (C.P.); 2 Department of Food Technology and Human Nutrition, Faculty of Biology and Agriculture, University of Rzeszów, 35-601 Rzeszów, Poland; ikapusta@ur.edu.pl (I.K.); jan.oszmianski@up.wroc.pl (J.O.); 3 Wrocław University of Environmental and Life Sciences, Faculty of Biotechnology and Food Science, Department of Fruit, Vegetable and Plant Nutraceutical Technology, 37 Chełmonskiego Street, 51-630 Wrocław, Poland

**Keywords:** water-based extraction, tea, magnetic field, chemical profile, polyphenols, caffeine

## Abstract

This article presents the findings of a study investigating the feasibility of using a magnetic field assisted technique for the water-based extraction of mineral components, polyphenols, and caffeine from dry black and green tea leaves. The authors present a concept of applying constant and variable magnetic fields in the process of producing water-based infusions from selected types of tea. Analyses investigating the effectiveness of the proposed technique in comparison with conventional infusion methods assessed the contents of selected mineral components—i.e., Al, Ca, Cu, K, Mg, P, S, and Zn—which were examined with the use of ICP-OES. The contents of caffeine and polyphenolic compounds were assessed using the HPLC. A changing magnetic field permitted an increased effectiveness of extraction of the mineral components, caffeine, and polyphenols. The findings support the conclusion that a changing magnetic field assisted extraction method is useful for obtaining biologically valuable components from tea infusions.

## 1. Introduction

Extraction is a method of separating certain components from a liquid or from a mixture of solids with the use of a solvent. The method is applied for instance in order to obtain natural substances from plant materials, such as tree bark, leaves, stems or even flowers. The growing demand for natural products observed in pharmaceutical, cosmetics, and—most importantly—food industry, has led to rapidly increasing interest in non-conventional extraction techniques, as a means of improving the effectiveness of the process [1]. Consequently nowadays, in addition to conventional water-based extraction with the use of higher temperatures or a longer duration of the process, researchers also explore less conventional methods such as supercritical carbon dioxide extraction [2]. Supercritical CO_2_ extraction was described in 1879 by Hannay and Hogarth, who showed that supercritical fluids were powerful solvents [3]. Yet, the method was not developed until 100 years later. The technique was applied, for instance, in the process of producing decaffeinated coffee and tea as well as in the extraction of hop essential oil [4].

In another model, extraction is facilitated by microwave radiation [5,6]. Microwave assisted extraction (MAE) uses the phenomenon of direct absorption of microwave radiation by particles of the substance, and its effectiveness results from the way thermal energy is transferred. Microwaves supply energy directly to a particle of a chemical component, with no loss of energy due to convection or conduction [7].

Nowadays, one of the most common methods applies ultrasound as an extraction enhancing factor [8,9]. The Ultrasound Assisted Extraction (UAE) technique takes advantage of the propagation of sound waves in liquids, which is associated with cycles of increased and decreased density, i.e., changes in pressure. Variable acoustic pressure results in secondary phenomena which promote the extraction process. A secondary phenomenon of major importance in the process of mass transfer is cavitation, a process of dynamic formation, growth, and collapse of vapor and gas cavities in a liquid. Ultrasound-assisted extraction applies low frequency acoustic oscillations, in the 20–50 kHz range, yet with a high intensity of 140–160 dB [10,11,12].

Less conventional methods include extraction mediated by superheated water [13], pulsed electric field [14,15], and electropermeabilization [16].

Seeking new ways to enhance extraction of bioactive substances from plant material, the authors of the present study applied extraction mediated by non-thermal constant magnetic field and non-thermal slowly-changing magnetic field. Black (fully fermented) and green (non-fermented) leaf teas were used as research materials. According to the literature, these two types of tea, if brewed (extracted) effectively, can provide protection against heart disease thanks to the active substances contained in them, and also reduce incidence of type 2 diabetes [17].

## 2. Results and Discussion

Extraction related issues have been described rather extensively in the literature along with tea infusion composition analyses focusing on particularly valuable substances [18,19,20]. The following analysis of the findings obtained during laboratory tests carried out with the use of permanent and slow-changing magnetic fields shows that various groups of substances respond in different ways to the magnetic field applied in the process of infusing.

Table 1 above shows that an increase in the concentrations of mineral components in the infusions was only linked with variable magnetic fields. It was observed that a variable magnetic field produced different effects in the extraction of selected metal ions from dry tea leaves to the various black tea infusions. Out of all the chemical elements, potassium was found to migrate most rapidly after a variable magnetic field was applied. In two out of the three tea brands, there was an over two-fold increase in the effectiveness of potassium ion extraction. A variable magnetic field assisted extraction also significantly improved the contents of Ca, Mg, and P ions in the final infusions of all the three tea brands.

The results showing mineral components extracted from the green tea (Table 2), just like those reported by Sembratowicz & Rusinek-Prystupa [21], confirm generally similar trends in mineral composition of green and black teas. Hence, tendencies corresponding to those identified in the black teas were also observed in the green teas with regard to extraction effectiveness induced by the additional factor, i.e., a magnetic field. In this case, a permanent magnetic field also failed to produce significant effects in the mineral composition of the infusion. Improved extraction was only observed after a variable magnetic field was applied, with the most effective extraction recorded in the case of calcium ions (with an improvement of up to 48%) and magnesium ions (increase in extraction effectiveness of up to 45%).

The most significant changes in extraction from both types of tea were observed when variable magnetic fields were applied, in particular in the case of magnesium, calcium, phosphorus, and potassium ions. Such ions may respond to external magnetic fields by seeking to either strengthen or weaken them, depending on their own magnetic structure. Additionally, a variable magnetic field may produce a resonance effect, changing the voltage of cell membranes in plant tissues, and by affecting a change of voltage on cell membranes it may lead to the more effective transport of substances via ion channels. The effects produced by magnetic fields in ion channels and the resulting transport of cations H^+^, Ca^2+^, and K^+^ were discussed by Levin [22]. Likewise, Huang, Ye, Xu, Liu, Qu [23] described the increased capacity for transporting Ca^2+^ ions into and out of cells as an effect of a sinusoidal magnetic field with a resonance frequency of 50 Hz.

Caffeine was another extracted active compound subjected to analyses (Table 3 and Table 4). Its content in the black teas extracted in a conventional way was in the range of 209.2–221.6 mg/L and in the green teas amounted to 243.2–244.7 mg/L.

Similar findings in these two groups of tea were reported by Hilal & Engelhardt [24], who used the HPLC technique to determine caffeine contents in three kinds of tea. After a constant magnetic field was applied, no statistically significant changes in caffeine contents were observed either in the black or green teas. On the other hand extraction mediated with a variable magnetic field produced a significant increase in caffeine contents in the final infusions. In the black teas, the change ranged from 3.6% to 12.1%, depending on the tea brand, and in the green teas there was an increase in the range from 5.9% to 17.5%.

Table 5 and Table 6 shown the level of polyphenols identified in the black and green tea infusions. The black teas were found with more varied contents of polyphenolic compounds in comparison with the green teas. Following application of a variable magnetic field there was an increase in the total contents of the polyphenols, yet no explicit tendencies were identified with respect to the specific compounds in this group of substances. On average the increase in the black teas amounted to 15% and in the green teas was at the level of 10%. Similar results were observed by Both, Chemat, and Strube [25]; and Wang, Zhao, Tian, Yan, and Guo [26] who applied an ultrasound assisted extraction technique. They reported a mean increase in the total contents of extracted polyphenols, in comparison to control samples, at the level of 15%. On the other hand, the use of a microwave assisted extraction technique, as described by Wang, Qin, and Hu [27] and Nkhili et al. [28] led to a 10% increase in polyphenol contents in the extract, but only at a temperature of 100 °C. The lower temperature used by these authors—i.e., 80 °C—failed to produce the same effect.

These results suggest that a magnetic field assisted extraction method could successfully be applied to enhance the effectiveness of the process of extracting the substances from tea leaves to the infusion. Most importantly, as a result it may be possible to design a ‘functional tea-based beverage’, similar to functional foods, producing physiological effects in the human body. Properly selected techniques designed to facilitate water-based extraction, mediated by ultrasound, microwaves, or magnetic fields as proposed here, and possibly applied in synergy, may lead to technological advancements in the extraction of bioactive substances from plant material.

## 3. Materials and Methods

### 3.1. Plant Material

Three tea brands were selected for each type (color) (Table 7).

### 3.2. Extraction Parameters

In each case, the extraction temperature was defined as 100 °C, whereby 100 mL of demineralized water was added to 2 g of tea; the entire process was carried out in flat-bottom flasks, with a diameter of 8 cm, tightly closed, with no mixing. The extraction process was conducted for the duration of five minutes in control conditions (C), with the use of permanent magnetic field assisted extraction (PMF) with an induction of 100 mT and with the use of variable magnetic field assisted extraction (VMF) with a frequency of 50 Hz and induction of 100 mT. Each extraction was performed in three independent repetitions. The permanent magnetic field was induced between a pair of neodymium magnets, positioned 10 cm apart. The stability of the magnetic field distribution is shown in Figure 1. The variable magnetic field was generated by an induction coil powered by an alternating current autotransformer. The stability of coil operation is shown in Figure 2.

### 3.3. Determination of Caffeine by HPLC Analysis

To determine caffeine contents, the infusions obtained were processed via MCE filters, with 0.45 μm pore size, and then diluted 100-fold. The analyses were performed with the use of a highly-efficient liquid chromatography system from YoungLin (Gyeonggi-do, Korea), consisting of a YL9110 quaternary pump with eluent mixer at low pressure, a YL9101 reagent vial coupled with vacuum phase degasser, a YL9131 thermostatted column, and a YL9120 UV–VIS detector. Chromatography separation was performed with the use of a Cosmosil 5C18-MS-II 4,6ID × 250 mm chromatography column with a SecurityGuard pre-column with C18 cartridge. Optimum parameters were determined for chromatography analysis, i.e., isocratic flow; composition of the mobile phase: water:methanol 70:30 *v*/*v*; speed of mobile phase flow: 0.6 cm^3^/min; injection volume: 20 μL; temperature inside the thermostatted column: 25 °C; duration of analysis: 25 min. The basic validation parameters were estimated by the applied analytic method. The specificity of the method was confirmed with model caffeine injections. Anhydrous caffeine (Caffeine Reference Standard) from Sigma-Aldrich was dissolved to prepare a model solution with defined concentration (1 g/dm^3^) and stored at 4 °C. This solution was the basis for preparing working model solutions (2, 4, 6, 8, 10 μg/cm^3^). Linearity of detector response was identified for the programmed concentrations of model solutions in the range from 2.0 to 10 μg/cm^3^ at 271 nm and UV2 201 nm wavelengths of UV1. The calibration curve obtained had a correlation coefficient (R2) of 0.999. The estimated yield, on average, amounted to 96.9% in the case of the black teas, and 97.4% in the green teas.

### 3.4. Determination of Mineral Content by ICP-OES Analysis

The composition of chemical elements in the infusions was determined using ICP-OES apparatus (Schaumburg, IL, USA), Thermo iCAP Dual 6500 with horizontal plasma, and capacity for detection along and across the plasma flame (radial and axial). Before measuring each batch of 10 samples, calibration was performed using certified (Merck) models, with concentrations of 10,000 ppm for Ca, Mg, K, P; and 1000 ppm for Al, Cu, S, Zn.

In each case a three-point calibration curve was used for each element, with optical adjustment applying the method of internal models, in the form of yttrium and ytterbium ions, at concentrations of 2 mg/L and 5 mg/L, respectively. The analytical methods were validated with two independent tests. Certified Reference Material (Tea leaves INCT-TL-1 and NIES CRM No. 7 Tea Leaves) was used and the recovery obtained for specific elements is shown in the Table 8 below. In order to identify the relevant measurement lines and avoid possible interferences, the method of adding a model with known concentration was applied (Environmental analysis, Method 200.7, US EPA, Drinking water).

### 3.5. Determination of Polyphenolic Compounds by HPLC MS Analysis

Polyphenolics were analyzed using the Waters ACQUITY system (Waters, Milford, MA, USA), consisting of a binary pump manager, sample manager, column manager, PDA detector, and tandem quadrupole mass spectrometer (TQD) with electrospray ionization (ESI). The separation was carried out using a BEH C18 column (100 × 2.1 mm i.d., 1.7 µm, Waters) kept at 50 °C. The following solvent system was applied: mobile phase A (0.1% formic acid in water *v*/*v*) and mobile phase B (0.1% formic acid in 40% ACN in water *v*/*v*). The gradient program was set as follows: 0 min 5% B, from 0 to 8 min linear to 100% B, and from 8 to 9.5 min for washing and back to initial conditions. The injection volume of the samples was 5 µL (partial loop with needle overfill) and the flow rate was 0.35 mL/min. The following parameters were used for TQD: capillary voltage 3.5 kV; con voltage 30 V in negative mode, the source was kept at 250 °C and the desolvation temperature was 350 °C; con gas flow 100 L/h; and desolvation gas flow 800 L/h. Argon was used as collision gas at a flow rate of 0.3 mL/min. The polyphenolics detection and identification being based on specific PDA spectra, mass-to-charge ratio and fragment ions obtained after collision induced dissociation (CID). All determinations were performed in duplicate. Waters MassLynx software v.4.1 was used for data acquisition and processing.

### 3.6. Statistical Analysis

The statistical hypotheses related to the effects of tea type and magnetic factor were verified with the use of two-way ANOVA with Tukey’s post-hoc test, at α = 0.05 and numbers of repetitions n = 3.

## 4. Conclusions

Statistical analyses showed slight differences in the contents of mineral components and caffeine in infusions of the relevant tea brands brewed in a conventional way. No improvement was identified in water-based extraction of any of the substances examined following application of a constant magnetic field; on the other hand, a significant improvement in extraction of the mineral substances and caffeine was observed when the process was facilitated by variable magnetic fields with induction of 100 mT and a frequency of 50 Hz. A small improvement was observed in the total content of polyphenols extracted using a variable magnetic field, yet various trends were recorded in the case of specific compounds in this group. It seems magneto-extraction based on the application of a variable magnetic field in the case of tea infusions may be a beneficial solution in assisting conventional water-based extraction techniques.

## Figures and Tables

**Figure 1:** Distribution of the permanent magnetic field, induction of *B* = 100 mT, within the sample subjected to extraction.

**Figure 2:** Distribution of variable magnetic field, induction of *B* = 100 mT and frequency of *f* = 50 Hz, within the sample subjected to extraction.

**Table 1:** Analytical findings showing contents of selected chemical elements in black tea infusions extracted with the use of a magnetic field under control conditions.

Tea	Factor	Mineral Content mg/L							
		Al	Ca	Cu	K	Mg	P	S	Zn
B1	C	5.41 ± 0.25 ^ab,^**	2.90 ± 0.12 ^a^	0.12 ± 0.05 ^a^	150 ± 8 ^a^	16.1 ± 1.9 ^ab^	52.2 ± 1.7 ^a^	20.1 ± 1.6 ^b^	0.92 ± 0.12 ^ab^
B1	PMF	5.02 ± 0.19 ^ab^	2.70 ± 0.15 ^a^	0.13 ± 0.02 ^a^	162 ± 10 ^a^	15.8 ± 1.7 ^ab^	55.6 ± 1.1 ^ab^	19.8 ± 1.1 ^b^	0.87 ± 0.09 ^a^
B1	VMF	6.10 ± 0.11 ^b^	4.01 ± 0.16 ^bc^	0.18 ± 0.03 ^ab^	380 ± 12 ^c^	22.3 ± 2.5 ^c^	60.2 ± 2.2 ^b^	26.3 ± 1.5 ^c^	0.99 ± 0.07 ^ab^
B2	C	4.90 ± 0.26 ^a^	4.11 ± 0.21 ^bc^	0.09 ± 0.02 ^a^	162 ± 10 ^a^	14.2 ± 1.5 ^a^	60.2 ± 2,1 ^b^	15.2 ± 1.2 ^a^	0.78 ± 0.11 ^a^
B2	PMF	5.02 ± 0.17 ^ab^	4.40 ± 0.18 ^c^	0.09 ± 0.04 ^a^	155 ± 14 ^a^	15.0 ± 1.8 ^ab^	60.1 ± 1.7 ^b^	15.2 ± 0.9 ^a^	0.77 ± 0.11 ^a^
B2	VMF	6.12 ± 0.08 ^b^	5.01 ± 0.07 ^d^	0.15 ± 0.06 ^a^	362 ± 13 ^c^	27.4 ± 1.5 ^c^	65.2 ± 1.2 ^c^	18.3 ± 0.5 ^b^	1.01 ± 0.07 ^ab^
B3	C	4.70 ± 0.21 ^a^	3.56 ± 0.22 ^b^	0.10 ± 0.04 ^a^	140 ± 11 ^a^	12.9 ^a^ ± 1.9	51.1 ± 0.9 ^a^	19.6 ± 1.1 ^b^	0.82 ± 0.15 ^a^
B3	PMF	5.02 ± 0.17 ^ab^	4.02 ± 0.11 ^bc^	0.11 ± 0.03 ^a^	142 ± 9 ^a^	12.3 ± 1.4 ^a^	50.2 ± 1.6 ^a^	19.2 ± 1.1 ^b^	0.88 ± 0.08 ^a^
B3	VMF	5.90 ± 0.19 ^b^	4.87 ± 0.14 ^d^	0.16 ± 0.05 ^a^	173 ± 12 ^ab^	25.2 ± 1.7 ^c^	56.3 ± 1.8 ^ab^	22.3 ± 1.2 ^bc^	0.90 ± 0.12 ^ab^

** Means with the same letter are not significantly different; α = 0.05 (Tukey’s test), n = 3.

**Table 2:** Analytical findings showing the content of selected chemical elements in green tea infusions extracted with the use of a magnetic field under control conditions.

Tea	Factor	Mineral Content, mg/L							
		Al	Ca	Cu	K	Mg	P	S	Zn
G1	C	7.11 ± 0.12 ^a^,**	5.07 ± 0.14 ^a^	0.16 ± 0.05 ^a^	465 ± 14 ^a^	31.0 ± 0.9 ^a^	68.2 ± 1.5 ^a^	26.5 ± 1.1 ^a^	0.95 ± 0.11 ^ab^
G1	PMF	7.21 ± 0.29 ^a^	5.02 ± 0.15 ^a^	0.15 ± 0.04 ^a^	450 ± 11 ^a^	32.2 ± 1.2 ^a^	67.5 ± 1.2 ^a^	26.1 ± 0.8 ^a^	0.97 ± 0.09 ^ab^
G1	VMF	7.98 ± 0.27 ^ab^	7.50 ± 0.07 ^c^	0.17 ± 0.02 ^ab^	511 ± 11 ^b^	45.2 ± 2.1 ^c^	80.1 ± 1.1 ^b^	29.1 ± 1.6 ^ab^	1.02 ± 0.05 ^ab^
G2	C	7.45 ± 0.19 ^a^	5.90 ± 0.20 ^ab^	0.15 ± 0.02 ^a^	470 ± 15 ^ab^	35.2 ± 1.5 ^ab^	70.0 ± 1.7 ^ab^	28.2 ± 1.4 ^ab^	0.90 ± 0.05 ^a^
G2	PMF	7.20 ± 0.25 ^a^	5.54 ± 0.29 ^a^	0.15 ± 0.03 ^a^	481 ± 14 ^ab^	34.2 ± 1.8 ^ab^	68.9 ± 1.5 ^a^	28.3 ± 1.0 ^ab^	0.91 ± 0.04 ^a^
G2	VMF	8.00 ± 0.22 ^ab^	6.87 ± 0.21 ^bc^	0.17 ± 0.02 ^ab^	551 ± 10 ^b^	48.7 ± 1.5 ^c^	82.1 ± 0.9 ^b^	28.7 ± 1.1 ^ab^	1.00 ± 0.07 ^ab^
G3	C	7.60 ± 0.26 ^a^	5.40 ± 0.22 ^a^	0.14 ± 0.03 ^a^	450 ± 15 ^a^	30.6 ± 1.2 ^a^	68.0 ± 1.3 ^a^	25.5 ± 1.3 ^a^	0.90 ± 0.10 ^a^
G3	PMF	7.52 ± 0.17 ^a^	5.21 ± 0.20 ^a^	0.12 ± 0.02 ^a^	455 ± 17 ^a^	31.0 ± 1.4 ^a^	68.2 ± 1.1 ^a^	25.0 ± 1.2 ^a^	0.90 ± 0.05 ^a^
G3	VMF	7.99 ± 0.09 ^ab^	7.10 ± 0.17 ^c^	0.14 ± 0.02 ^a^	550 ± 10 ^b^	42.1 ± 1.5 ^bc^	79.3 ± 1.4 ^b^	29.1 ± 1.7 ^ab^	0.96 ± 0.07 ^ab^

** Means with the same letter are not significantly different; α = 0.05 (Tukey’s test), n = 3.

**Table 3:** Analytical findings showing contents of caffeine in black tea infusions extracted with the use of a magnetic field under control conditions.

Tea	Factor	Caffeine, mg/L
B1	C	217.7 ± 3.9 ^a,^**
B1	PMF	215.9 ± 3.1 ^a^
B1	VMF	228.2 ± 2.5 ^b^
B2	C	209.2 ± 3.7 ^a^
B2	PMF	209.5 ± 4.9 ^a^
B2	VMF	216.7 ± 3.7 ^a^
B3	C	221.6 ± 2.9 ^ab^
B3	PMF	225.6 ± 2.7 ^ab^
B3	VMF	248.4 ± 2.2 ^c^

** Means with the same letter are not significantly different; α = 0.05 (Tukey’s test), n = 3.

**Table 4:** Analytical findings showing contents of caffeine in green tea infusions extracted with the use of a magnetic field under control conditions.

Tea	Factor	Caffeine, mg/L
G1	C	244.6 ± 5.9 ^ab^ **
G1	PMF	241.2 ± 5.1 ^ab^
G1	VMF	287.3 ± 2.1 ^c^
G2	C	234.2 ± 1.9 ^a^
G2	PMF	240.6 ± 3.6 ^ab^
G2	VMF	271.3 ± 2.2 ^c^
G3	C	247.7 ± 2.5 ^ab^
G3	PMF	250.1 ± 3.7 ^b^
G3	VMF	262.2 ± 4.9 ^b^

** Means with the same letter are not significantly different; α = 0.05 (Tukey’s test), n = 3.

**Table 5:** Analytical findings showing contents of selected polyphenolic compounds in black tea infusions extracted with the use of a magnetic field under control conditions.

Tea	Factor	Polyphenolic Compounds mg/mL																	
		1 *	2	3	4	5	6	7	8	9	10	11	12	13	14	15	16	17	Total
B1	C	0.054 ± 0.011	0.021 ± 0.003	0.014 ± 0.002	0.022 ± 0.005	0.059 ± 0.012	0.118 ± 0.012	0.040 ± 0.003	0.080 ± 0.005	0.032 ± 0.004	0.061 ± 0.005	0.036 ± 0.003	0.169 ± 0.015	0.049 ± 0.005	0.077 ± 0.003	0.045 ± 0.003	0.071 ± 0.002	0.028 ± 0.004	0.976 ^b,^**
B1	PMF	0.056 ± 0.009	0.022 ± 0.005	0.014 ± 0.002	0.021 ± 0.005	0.058 ± 0.009	0.098 ± 0.009	0.048 ± 0.003	0.080 ± 0.007	0.033 ± 0.004	0.063 ± 0.011	0.029 ± 0.004	0.178 ± 0.016	0.058 ± 0.005	0.086 ± 0.004	0.049 ± 0.004	0.065 ± 0.006	0.032 ± 0.004	0.990 ^b^
B1	VMF	0.056 ± 0.007	0.026 ± 0.005	0.015 ± 0.003	0.022 ± 0.004	0.061 ± 0.008	0.136 ± 0.015	0.046 ± 0.006	0.083 ± 0.004	0.036 ± 0.002	0.064 ± 0.006	0.034 ± 0.004	0.198 ± 0.014	0.067 ± 0.004	0.093 ± 0.003	0.046 ± 0.004	0.082 ± 0.004	0.039 ± 0.005	1.103 ^c^
B2	C	0.045 ± 0.005	0.020 ± 0.003	0.011 ± 0.002	0.019 ± 0.001	0.054 ± 0.011	0.089 ± 0.009	0.047 ± 0.005	0.081 ± 0.010	0.023 ± 0.002	0.062 ± 0.004	0.019 ± 0.002	0.187 ± 0.022	0.055 ± 0.005	0.084 ± 0.006	0.041 ± 0.004	0.063 ± 0.005	0.030 ± 0.003	0.930 ^b^
B2	PMF	0.052 ± 0.005	0.020 ± 0.004	0.012 ± 0.004	0.022 ± 0.002	0.059 ± 0.008	0.115 ± 0.008	0.040 ± 0.011	0.080 ± 0.009	0.032 ± 0.004	0.051 ± 0.004	0.016 ± 0.002	0.169 ± 0.009	0.049 ± 0.007	0.077 ± 0.008	0.039 ± 0.005	0.066 ± 0.004	0.032 ± 0.001	0.931 ^b^
B2	VMF	0.055 ± 0.004	0.028 ± 0.008	0.011 ± 0.005	0.032 ± 0.003	0.087 ± 0.007	0.145 ± 0.014	0.050 ± 0.007	0.078 ± 0.004	0.035 ± 0.002	0.062 ± 0.005	0.032 ± 0.004	0.189 ± 0.016	0.059 ± 0.006	0.099 ± 0.007	0.042 ± 0.004	0.081 ± 0.006	0.033 ± 0.002	1.118 ^c^
B3	C	0.023 ± 0.012	0.019 ± 0.004	0.008 ± 0.003	0.018 ± 0.004	0.041 ± 0.011	0.078 ± 0.009	0.044 ± 0.007	0.080 ± 0.005	0.019 ± 0.002	0.052 ± 0.005	0.017 ± 0.002	0.145 ± 0.011	0.054 ± 0.004	0.045 ± 0.005	0.023 ± 0.002	0.062 ± 0.007	0.029 ± 0.004	0.757 ^a^
B3	PMF	0.024 ± 0.005	0.020 ± 0.005	0.007 ± 0.002	0.019 ± 0.006	0.055 ± 0.005	0.077 ± 0.003	0.039 ± 0.005	0.070 ± 0.006	0.023 ± 0.003	0.044 ± 0.005	0.016 ± 0.001	0.132 ± 0.012	0.041 ± 0.007	0.044 ± 0.005	0.021 ± 0.002	0.072 ± 0.005	0.036 ± 0.004	0.740 ^a^
B3	VMF	0.030 ± 0.006	0.030 ± 0.006	0.009 ± 0.001	0.030 ± 0.006	0.065 ± 0.012	0.080 ± 0.005	0.044 ± 0.006	0.081 ± 0.006	0.023 ± 0.004	0.041 ± 0.003	0.018 ± 0.004	0.154 ± 0.012	0.049 ± 0.008	0.040 ± 0.003	0.042 ± 0.006	0.078 ± 0.009	0.039 ± 0.006	0.853 ^b^

** Means with the same letter are not significantly different; α = 0.05 (Tukey’s test), n = 3. * **1**—neochlorogenic acid; **2**—Trigalloyl glucose; **3**—(−)epigallocatechin; **4**—coumaroyl-quinic acid; **5**—3-coumaroyl-quinic acid; **6**—chlorogenic acid; **7**—4-coumaroyl-quinic acid; **8**—5-coumaroyl-quinic acid; **9**—Kaempferol-*O*-rhamnosyl-*O*-pentoside; **10**—Kaempferol-3-*O*-sophoroside-7-*O*-glucoside; **11**—Kaempferol-3-*O*-rhamnosyl-galactoside; **12**—Quercetin-3-*O*-rutinoside; **13**—epigallocatechin-3-gallate; **14**—Quercetin-3-*O*-glucoside; **15**—Kaempferol-3-*O*-rutinoside-7-*O*-galactoside; **16**—Kaempferol-3-*O*-rhamnosyl-galactoside; **17**—Kaempferol-3-*O*-glucoside.

**Table 6:** Analytical findings showing contents of selected polyphenolic compounds in green tea infusions extracted with the use of a magnetic field under control conditions

Tea	Factor	Polyphenolic Compounds mg/mL																	
		1 *	2	3	4	5	6	7	8	9	10	11	12	13	14	15	16	**17**	**Total**
G1	C	0.026 ± 0.003	0.026 ± 0.005	nd	0.127 ± 0.011	nd	0.053 ± 0.005	nd	nd	0.034 ± 0.002	0.070 ± 0.006	0.022 ± 0.003	0.105 ± 0.009	0.010 ± 0.002	0.064 ± 0.006	0.120 ± 0.006	0.102 ± 0.008	0.103 ± 0.006	0.862 ^b,^**
G1	PMF	0.029 ± 0.004	0.027 ± 0.002	nd	0.154 ± 0.012	nd	0.068 ± 0.006	nd	nd	0.032 ± 0.003	0.066 ± 0.003	0.031 ± 0.002	0.098 ± 0.007	0.017 ± 0.003	0.060 ± 0.005	0.116 ± 0.006	0.090 ± 0.008	0.093 ± 0.007	0.882 ^bc^
G1	VMF	0.029 ± 0.004	0.031 ± 0.001	nd	0.146 ± 0.009	nd	0.063 ± 0.007	nd	nd	0.043 ± 0.003	0.087 ± 0.005	0.026 ± 0.002	0.102 ± 0.005	0.025 ± 0.002	0.069 ± 0.006	0.112 ± 0.009	0.124 ± 0.011	0.130 ± 0.011	0.987 ^c^
G2	C	0.022 ± 0.006	0.024 ± 0.002	nd	0.117 ± 0.008	nd	0.051 ± 0.005	nd	nd	0.032 ± 0.002	0.066 ± 0.005	0.024 ± 0.001	0.109 ± 0.005	0.012 ± 0.002	0.052 ± 0.003	0.112 ± 0.014	0.099 ± 0.006	0.101 ± 0.014	0.821 ^b^
G2	PMF	0.027 ± 0.004	0.023 ± 0.004	nd	0.114 ± 0.012	nd	0.055 ± 0.002	nd	nd	0.031 ± 0.004	0.059 ± 0.007	0.024 ± 0.002	0.102 ± 0.006	0.013 ± 0.004	0.059 ± 0.003	0.121 ± 0.009	0.089 ± 0.007	0.099 ± 0.012	0.816 ^b^
G2	VMF	0.032 ± 0.006	0.036 ± 0.007	nd	0.132 ± 0.015	nd	0.087 ± 0.003	nd	nd	0.055 ± 0.002	0.087 ± 0.008	0.021 ± 0.003	0.087 ± 0.008	0.009 ± 0.001	0.045 ± 0.001	0.098 ± 0.011	0.082 ± 0.006	0.089 ± 0.011	0.860 ^bc^
G3	C	0.019 ± 0.005	0.019 ± 0.002	nd	0.109 ± 0.007	nd	0.045 ± 0.003	nd	nd	0.021 ± 0.005	0.059 ± 0.006	0.026 ± 0.002	0.101 ± 0.012	0.011 ± 0.002	0.042 ± 0.004	0.118 ± 0.009	0.087 ± 0.007	0.105 ± 0.009	0.762 ^a^
G3	PMF	0.018 ± 0.004	0.018 ± 0.002	nd	0.114 ± 0.006	nd	0.044 ± 0.004	nd	nd	0.020 ± 0.004	0.051 ± 0.005	0.021 ± 0.005	0.105 ± 0.011	0.011 ± 0.004	0.042 ± 0.003	0.102 ± 0.008	0.098 ± 0.009	0.102 ± 0.008	0.746 ^a^
G3	VMF	0.036 ± 0.002	0.042 ± 0.004	nd	0.126 ± 0.009	nd	0.078 ± 0.004	nd	nd	0.042 ± 0.001	0.060 ± 0.004	0.014 ± 0.002	0.099 ± 0.009	0.012 ± 0.001	0.056 ± 0.004	0.098 ± 0.007	0.092 ± 0.004	0.098 ± 0.008	0.853 ^b^

** Means with the same letter are not significantly different; α = 0.05 (Tukey’s test), n = 3; nd—not detected. * **1**—neochlorogenic acid; **2**—Trigalloylglucose; **3**—(−)epigallocatechin; **4**—coumaroyl-quinic acid; **5**—3-coumaroyl-quinic acid; **6**—chlorogenic acid; **7**—4-coumaroyl-quinic acid; **8**—5-coumaroyl-quinic acid; **9**—Kaempferol-*O*-rhamnosyl-*O*-pentoside; **10**—Kaempferol-3-*O*-sophoroside-7-*O*-glucoside; **11**—Kaempferol-3-*O*-rhamnosyl-galactoside; **12**—Quercetin-3-*O*-rutinoside; **13**—epigallocatechin-3-gallate; **14**—Quercetin-3-*O*-glucoside; **15**—Kaempferol-3-*O*-rutinoside-7-*O*-galactoside; **16**—Kaempferol-3-*O*-rhamnosyl-galactoside; **17**—Kaempferol-3-*O*-glucoside.

**Table 7:** List of tea brands selected for laboratory analyses.

Name	Symbol Used in the Article	Country of Origin	Tea Color
Sencha	G1	Japan	Green
Gyokuro	G2	Japan	Green
Bancha	G3	Japan	Green
English Breakfast	B1	Sri-Lanka	Black
Darjeeling	B2	India	Black
Yunnan	B3	China	Black

**Table 8:** Measurements parameters and recovery for specific elements.

Element	Measurement Line, nm	Recovery According to CRM, %	Recovery According to Known Addition Method, %
Al	167.079	98	100
Ca	317.933	101	99
Cu	324.754	98	99
K	766.490	102	98
Mg	279.533	102	101
P	177.495	101	99
S	180.731	97	100
Zn	213.856	99	97

The detection limit for each element was determined at a level which was not lower than 1 µg/L.
